This article has been retracted.

# Heavy metal accumulation by roadside vegetation and implications for pollution control

**DOI:** 10.1371/journal.pone.0249147

**Published:** 2021-05-13

**Authors:** Rubina Altaf, Sikandar Altaf, Mumtaz Hussain, Rahmat Ullah Shah, Rehmat Ullah, Muhammad Ihsan Ullah, Abdul Rauf, Mohammad Javed Ansari, Sulaiman Ali Alharbi, Saleh Alfarraj, Rahul Datta

**Affiliations:** 1 Department of Botany, University of Agriculture Faisalabad, Faisalabad, Punjab, Pakistan; 2 Institute of Environmental Science and Engineering, School of Civil and Environmental Engineering, National University of Science and Technology, Islamabad, Pakistan; 3 Department of Soil Science, Faculty of Agricultural Sciences and Technology, Bahauddin Zakariya University, Multan, Pakistan; 4 Soil and Water Testing Laboratory, Dera Ghazi Khan, Pakistan; 5 Sorghum Research Substation, Department of Agriculture, Dera Ghazi Khan, Pakistan; 6 Department of Agricultural Research (Field), Dera Ghazi Khan, Pakistan; 7 Department of Botany, Hindu College Moradabad (Mahatma Jyotiba Phule Rohilkhand University Bareilly), Moradabad, India; 8 Department of Botany & Microbiology, College of Science, King Saud University, Riyadh, Saudi Arabia; 9 Zoology Department, College of Science, King Saud University, Riyadh, Saudi Arabia; 10 Department of Geology and Soil Science, Faculty of Forestry and Wood Technology, Mendel University in Brno, Brno, Czech Republic; Harran Üniversitesi: Harran Universitesi, TURKEY

## Abstract

Vehicular emissions cause heavy metal pollution and exert negative impacts on environment and roadside vegetation. Wild plants growing along roadsides are capable of absorbing considerable amounts of heavy metals; thus, could be helpful in reducing heavy metal pollution. Therefore, current study inferred heavy metal absorbance capacity of some wild plant species growing along roadside. Four different wild plant species, i.e., *Acacia nilotica* L., *Calotropis procera* L., *Ricinus communis* L., and *Ziziphus mauritiana* L. were selected for the study. Leaf samples of these species were collected from four different sites, i.e., Control, New Lahore, Nawababad and Fatehabad. Leaf samples were analyzed to determine Pb^2+^, Zn^2+^, Ni^2+^, Mn^2+^ and Fe^3+^ accumulation. The *A*. *nilotica*, *Z*. *mauritiana* and *C*. *procera* accumulated significant amount of Pb at New Lahore site. Similarly, *R*. *communis* and *A*. *nilotica* accumulated higher amounts of Mn, Zn and Fe at Nawababad and New Lahore sites compared to the rest of the species. Nonetheless, *Z*. *mauritiana* accumulated higher amounts of Ni at all sites compared with the other species included in the study. Soil surface contributed towards the uptake of heavy metals in leaves; therefore, wild plant species should be grown near the roadsides to control heavy metals pollution. Results revealed that wild plants growing along roadsides accumulate significant amounts of heavy metals. Therefore, these species could be used to halt the vehicular pollution along roadsides and other polluted areas.

## Introduction

Environmental pollution harms earth’s ecosystems due to toxic substances and energy release into air, land and water. Air pollution is the most noxious among all of the pollution types [1–5]. Vehicular emission is a significant source of air pollution. Heavy metals like iron (Fe), cadmium (Cd), lead (Pb), copper (Cu), chromium (Cr), nickel (Ni), zinc (Zn) and manganese (Mn) are released from several wires, alloy, tires and pipes of vehicles into roadside surroundings [6–10]. Motor vehicles are regarded as the main source of air pollution globally. Motor vehicles release carbon monoxide, the major part of nitrogen oxides (NOx), volatile organic compounds (VOCs), toxic chemicals and some fine particles [11–14]. The sources of heavy metals include leather tanning, lead-acid batteries, fluorescent, fuel, battery industry and thermal power plants [15].

Heavy metals such as Fe, Cu, Ni, Cd, Cu, Pb and Zn are released through different parts of vehicles [16–20]. Heavy metals emitted from various sources are accumulated on the soil surface [18, 21, 22]. Human activities are the main cause of heavy metal pollution [17, 23, 24]. Every year, millions of tons of heavy metals are released into the air, which destroy environmental ecology and ecosystem and negatively affect human health [25–30].

The effects of vehicular pollution appear on the physiological aspects of plants [31–34]. The pH of soil is gradually altered by the absorption of heavy metals that affect anatomical, physiological and reproductive attributes of plants [35–38]. Reproductive parts of plants are adversely affected by automobile’s emission [38–40]. Heavy metal pollution affects seedling growth and germination of roadside vegetation [41–43]. The germination rate of seeds is decreases due to excessive Pb toxicity [44, 45]. Remediation is mandatory to control heavy metal pollution for recovery and restoration of ecosystem [46, 47]. Many remediation technologies have been developed to avoid the harmful effects of heavy metal pollution. Phytoremediation is a low cost and highly useful technique for the reduction of heavy metals’ pollution. Different types of plants with high absorbance capacity for heavy metals can be used in phytoremediation [48–50].

Different plant species are known to absorb, detoxify and tolerate higher levels of heavy metal pollution [51, 52]. Few tree species, including *Mangifera indica* L., *Pongamia pinnata* L. Pierre, *Dalbergia sissoo* Roxb and *Holoptelea integrifolia* L. are used to control air pollutants [53–55]. Roadside plants are usually more tolerant to heavy metals and indicate their competent capability for plantation in ecological areas for urban ecosystem restoration [26, 56]. The rate of urbanization in Pakistan is about 38.6%. Therefore, roads loaded with high traffic produce higher amounts of heavy metal pollution. Pakistan is trying to control vehicular pollution with limited resources and awareness [57].

Vegetation and soil samples are the most economical and easiest ways to assess heavy metals’ pollution in roadsides [58–60], some other plants [61, 62], grasses [63] and few other organisms like fish [64, 65] have been used to monitor heavy metal pollution. Due to relative importance of wild plants and places, current study was conducted to infer heavy metal accumulation capacity of different wild species growing along roadsides. The particular objectives of the study were; i) to investigate the concentration of selected heavy metals in the leaves of different wild plants at different sites, ii) to compare the amount of heavy metals between plants and sites and iii) to estimate the concentration of heavy metals in soil from selected sites. The results will help to select the plants for phytoremediation purposes along roadsides.

## Materials and methods

### Plant species

Four plant species, i.e., *Acacia nilotica* L., *Calotropis procera* L., *Ricinus communis* L. and *Ziziphus mauritiana* Lam. were selected for the current study.

### Collection of plant samples

The leaves of these species were collected from four different sites, i.e., control, New Lahore, Nawababad and Fatehabad. Control site was selected 50 meters away from the roadside to exclude the risk of vehicular emission. The plant leaves were cut with a cutter, sealed in polythene bags and brought to the laboratory for further analysis.

### Determination of heavy metals in leaf samples

For evaluating heavy metal accumulation, leaf samples were dried in an oven at 70°C for 15 days. The digestion process was used following [66, 67] for the estimation of heavy metal accumulation.

### Digestion method

The 0.1g of dried plant leaves were added in a conical digestion flask, where 6ml of Nitric acid (HNO_3_) was added and kept overnight at 25°C. Digestion flask was placed on the hot plate at 150°C until the acid evaporated. When fumes appeared, 1ml hydrogen peroxide (H_2_O_2_) was added to each digestion flask. Then sample flask was left to cool down, and the colorless liquid solution was diluted by measuring the flask with 50 ml water. The filtered solution was used to measure heavy metals (Pb^2+^, Zn^2+^, Ni^2+^, Mn^2+,^ and Fe^3+^) accumulation using Atomic Absorption Spectrophotometer (Perkin Elmer) [68, 69].

### Soil sampling and determination of heavy metals in soil samples

The soil samples were collected from selected sites. The 500 g of soil was collected from each site and stored in polythene bags. The sample preparation method was identical, as mentioned above, to evaluate heavy metals concentration in soil samples.

### Determination of soil pH and Electrical Conductivity (EC)

The soil samples (200 g) were collected from each study site. soil paste made by gradual addition of distilled water to the samples with the help of a spatula. There was no free water on the surface of the paste. The paste was kept for saturation and distilled water was added according to the needs. The mixture was held for 16 hours. Filtration was done using a Vacuum filtration system with the Buchner funnel having a filter paper. The filtrate was collected in glass bottles and analyzed. The pH of the soil was determined by using a pH meter. The EC of soil was determined by using an EC meter [70].

### Physiological parameters

#### Determination of chlorophyll and carotenoid contents

The chlorophyll a, b, total chlorophyll, and carotenoids contents were determined according to the method of [71, 72]. Fresh leaves were cut into small pieces and placed into 5 ml of 80% acetone solution. The solution was filtered and centrifuged at 14000 rpm for 15 minutes at 4°C. The absorbance was calculated at 663 nm (chlorophyll b), 645 nm (chlorophyll a) and 480 nm (carotenoids) using a spectrophotometer (Hitachi Model U2800 Japan). The chlorophyll and carotenoids substances were obtained by following formulas 1, 2, and 3, respectively.

### Chlorophyll a

*Chl a (mg/g*^*-1*^ *leaf fresh weight) = [12*.*7(OD 663)– 2*.69 (OD 645)] * V/1000 * W.

### Chlorophyll b

*Chl b (mg/g*^*-1*^ *leaf fresh weight) = [22*.*9 (OD 645)– 4*.68 (OD 663)] * V/1000 * W.

### Total chlorophyll

*Total chl (mg/g*^*-1*^ *leaf fresh weight) = [20*.*2 (OD 645)– 8*.02 (OD 663)] * V/1000 * W.

### Carotenoids

*Carotenoids (mg/g*^*-1*^ leaf fresh weight) = [Acar/EM] * V/1000 * W.
*Acar = OD 480+ 0*.*114 (OD 663)– 0*.*638 (OD 645)*
Where, EM = 100% = 2500, OD = Optical density = Volume of sample and W = Weight of sample.

### Statistical analysis

The collected data were analyzed using one-way analysis of variance (ANOVA). Means were compared using Duncan Multiple Range Test (DMR) where ANOVA indicated significant differences [73, 74].

## Results

### Manganese accumulation

The highest concentration of Mn (1.1 mg/g) was noted in *A*. *nilotica* compared with other three wild plants (Fig 1A). The mean Mn concentration significantly varied among plants and sites. The lowest Mn (0–0.1 mg/g) was accumulated at control site. The Mn concentration was high (1.43 mg/g) in *R*. *communis* at New Lahore site, while at Nawababad site higher Mn accumulation (1.6 mg/g) was noted for *A*. *nilotica*. On the other hand, at sites 1 and 2, Mn accumulation was high (Fig 1C), and at site 2, a higher concentration was obtained in all plant species (Table 1). Table 1 illustrated mean values, which could be higher significant differences of Mn for the *Acacia nilotica* and *Ricinus communis* from Nawababad. The lowest amount of Mn in the leaves was estimated at control site, which significantly differed from all other sites. Overall, *A*. *nilotica* and *R*. *communis* accumulated the highest amounts of Mn.

**Fig 1:** Heavy metal accumulation in different wild plant species growing on roadside in a heavy automobile emission area, means sharing same letters are statistically non-significant (p>0.05).

**Table 1:** Interactive effect of wild plants and sites on accumulation of different metals in the leaves of studied plant species.

Sites	Plants	Mn (mg g^-1^)	Pb (mg g^-1^)	Zn (mg g^-1^)	Ni (mg g^-1^)	Fe (mg g^-1^)
**Control**	*A*. *nilotica*	0.13 c	1.16 e	0.09 d	1.12 f	0.21 f
	*C*. *procera*	1.31 ab	4.42 cd	1.88 a	6.28 c	2.44 a
	*R*. *communis*	1.59 a	4.54 bcd	1.42 b	6.37 bc	2.47 a
	*Z*. *mauritiana*	1.39 ab	4.86 bc	1.92 a	6.35 bc	2.46 a
**New Lahore**	*A*. *nilotica*	0.20 c	1.18 e	0.09 d	0.07 f	0.47 e
	*C*. *procera*	1.24 b	4.92 b	1.94 a	6.27 c	1.49 d
	*R*. *communis*	1.40 ab	4.28 d	1.94 a	6.50 abc	1.49 d
	*Z*. *mauritiana*	1.31 ab	4.75 bcd	1.91 a	6.35 bc	1.49 d
**Nawababad**	*A*. *nilotica*	0.07 c	1.23 e	0.05 d	0.72 e	0.48 e
	*C*. *procera*	1.40 ab	4.72 bcd	1.18 bc	6.13 c	1.49 d
	*R*. *communis*	1.56 a	4.48 bcd	1.43 b	6.19 c	1.45 d
	*Z*. *mauritiana*	1.14 b	4.58 bcd	1.70 a	6.29 c	1.46 d
**Fatehabad**	*A*. *nilotica*	0.08 c	1.13 e	0.10 d	0.95 de	0.49 e
	*C*. *procera*	1.12 b	5.64 a	1.39 bc	6.68 ab	1.70 c
	*R*. *communis*	1.16 b	4.83 bc	1.17 c	6.85 a	1.66 c
	*Z*. *mauritiana*	1.18 b	4.72 bcd	1.39 bc	6.66 ab	1.88 b
***LSD 0*.*05***		0.29	0.48	0.24	0.37	0.07

Means sharing same letters within a column are statistically non-significant (p>0.05).

### Lead accumulation

The highest Pb accumulation was recorded for *Z*. *mauritiana*, while the lowest Pb was accumulated by *A*. *nilotica* (Fig 1B). At New Lahore, the highest amount of Pb (6 mg/g) was recorded in *Z*. *mauritiana* than all other plants and sites (Table 1). *A*. *nilotica* has been reported as a good indicator of roadside pollution. The new Lahore site has heavy traffic, which possibly emit significant amounts of Pb. Therefore, *A*. *nilotica* accumulated higher Pb at this site. Plants by sites interaction indicated that Pb concentration differed among plants at various sites. The highest Pb was acquired by *Z*. *mauritiana* (5.638 mg/g) at New Lahore site followed by *C*. *procera* at New Lahore and *A*. *nilotica* at Fatehabad site (Table 1).

### Zinc accumulation

The lowest amount of Zn was accumulated by *Z*. *mauritiana*, while *C*. *procera* accumulated higher amount (1.10 mg/g) of Zn (Fig 1C). Higher Zn was present in soil at New Lahore and Fatehabad sites (1.5 and 1.9 mg/g) than other sites. *A*. *nilotica*, *C*. *procera* and *Z*. *mauritiana* accumulated significant amount of Zn at site 2 (Fig 3D). Plant by sites interaction demonstrated the four different levels for comparison (Table 1). *R*. *communis* accumulated lower Zn level than *A*. *nilotica* and *C*. *procera*. Similarly, *A*. *nilotica* acquired less Zn than *C*. *procera* at New Lahore site, while a higher Zn amount was observed in *C*. *procera* at Nawababad site (Table 1).

### Nickel accumulation

The increased concentration of Ni was recorded for *Z*. *mauritiana*, whereas the lowest amount of Ni was noted for *R*. *communis* (Fig 1D). The Ni (6–7 mg/g) was accumulated by tested plants at all sites except control. The Ni accumulation was in the order *Z*. *mauritiana*, *C*. *procera*, *A*. *nilotica* and *R*. *communis* (Fig 1D). The results revealed that *Z*. *mauritiana* found appropriate for decreasing Ni pollution.

### Iron accumulation

*A*. *nilotica* absorbed the highest concentration of Fe, while *R*. *communis* accumulated the lowest amount of Fe (Fig 2). Soil samples indicated that all sites had deposited increased amount of Fe (Fig 2). On the other hand, *A*. *nilotica* absorbed the highest concentration of Fe at New Lahore site (Table 1) than other sites. *C*. *procera* and *R*. *communis* accumulated same amount of Fe, while *A*. *nilotica* differed from the rest of the plant species.

**Fig 2:** Iron accumulation in in different wild plant species growing on roadside in a heavy automobile emission area, means sharing same letters are statistically non-significant (p>0.05).

### Heavy metal accumulation in soil

The physicochemical properties of soil samples collected from the study sites are shown in Table 2. The pH of the soil samples was alkaline, which varied among sites. The EC values were almost similar to earlier studies [75]. Soils had higher concentrations of Pb and Ni compared to other heavy metals (Fig 3). Similarly, some researchers [76, 77] examined heavy metal accumulation in the soil. The Pb and Ni are extensively released metals from the exhaust of vehicles. High concentrations of these metals is linked with high EC as EC can directly affect the availability of ions in the soil. The saline nature of the soil represented the high EC values. The level of other heavy metals except Pb and Ni in soil samples was low. Because of alkaline pH, soil induced metal ions retention and immobilization [78]. This is also possible due to the limited effect of leaching in the soil nutrients [79].

**Fig 3:** Heavy metal concentrations (mg/g dry weight) in the soil at various sites along Faisalabad-Jhang road.

**Table 2:** Basic physicochemical parameters of the soil samples for selected different sites.

Sites	pH	EC (μs/m)
Control	6.88 ± 0.21	13.71 ± 0.71
New Lahore	7.18 ± 0.05	26.36 ± 1.90
Nawababad	8.19 ± 0.12	27.73 ± 1.88
Fatehabad	8.47 ± 0.27	27.46 ± 1.29

Means sharing same letters within a column are statistically non-significant (p>0.05).

### Effect of heavy metals on physiological parameters

#### Chlorophyll a

Chlorophyll a content was higher in *A*. *nilotica* and *C*. *procera* than other plant species (Fig 4A). Chlorophyll a concentration was increased by 3 mg/g in *C*. *procera* at control site, while lower at other sites (Table 3). The highest chlorophyll a was noted in *C*. *procera* at control site, while *A*. *nilotica*, *R*. *communis* and *Z*. *mauritiana* concentration level was lower at Fatehabad site (Table 3).

**Fig 4:** Physiological attributes of different wild plant species growing on roadside in a heavy automobile emission area.

**Table 3:** Interactive effect of wild plants and sites on different biochemical parameters of studied plant species.

Sites	Plants	Chlorophyll a (mg g^-1^)	Chlorophyll b (mg g^-1^)	Carotenoids (mg g^-1^)	Total chlorophyll (mg g^-1^)
**Control**	*A*. *nilotica*	2.09 b	3.03 ab	5.01 a	4.05 a
	*C*. *procera*	1.59 bc	1.26 c	1.27 d	1.14 c
	*R*. *communis*	1.25 bc	1.27 c	1.31 d	1.25 c
	*Z*. *mauritiana*	1.55 bc	1.35 c	1.27 d	1.39 c
**New Lahore**	*A*. *nilotica*	3.07 a	3.72 a	4.01 b	4.12 a
	*C*. *procera*	1.14 c	1.21 c	1.16 d	1.18 c
	*R*. *communis*	1.13 c	1.24 c	1.13 d	1.30 c
	*Z*. *mauritiana*	1.14 c	1.17 c	1.14 d	1.32 c
**Nawababad**	*A*. *nilotica*	2.07 b	2.40 b	3.03 c	3.41 b
	*C*. *procera*	1.13 c	1.24 c	1.11 d	1.30 c
	*R*. *communis*	1.17 c	1.18 c	1.18 d	1.20 c
	*Z*. *mauritiana*	1.11 c	1.18 c	1.14 d	1.30 c
**Fatehabad**	*A*. *nilotica*	2.11 b	2.75 b	1.68 d	3.05 ab
	*C*. *procera*	1.34 bc	1.30 c	1.18 d	1.33 c
	*R*. *communis*	1.53 bc	1.17 c	1.28 d	1.36 c
	*Z*. *mauritiana*	1.41 bc	1.30 c	1.23 d	1.34 c
***LSD 0*.*05***		0.087	0.082	0.76	0.75

Means sharing same letters within a column are statistically non-significant (p>0.05).

#### Chlorophyll b

The higher amount of chlorophyll b was measured for *C*. *procera* with 1.8 mg/g, and 1.4 mg/g of chlorophyll b was recorded from *R*. *communis* (Fig 4B). Chlorophyll b in was lower at all sites in all plants except control site. Besides, chlorophyll b amount at all site was lower than control site (Table 3). Similarly, in all plant species concentration of chlorophyll b was highest at the control site as compared to all other sites (Table 3).

#### Total chlorophyll

Total chlorophyll concentration was lowest in *R*. *communis* and *Z*. *mauritiana* (Fig 4D). All plant species accumulated higher total chlorophyll content at control site than rest of the sites (Table 3). Total chlorophyll concentration at control site was 3.6 mg/g, while it was lower at all other sites. The lower total chlorophyll was found in all plant species at all sites except control (Table 3).

#### Carotenoids

The carotenoids content in different plants were *A*. *nilootica* ˃ *C*. *procera* ˃ *R*. *communis* ˃ *Z*. *mauritiana* (Fig 4C). Similarly, carotenoids content in leaf samples of all plants followed the order control ˃ New Lahore ˃ Nawababad ˃ Fatehabad (Table 3). Regarding sites, lower carotenoids contents were found at all sites than control site.

## Discussion

The experimental analysis conducted by Anwar et al. [80] revealed that some heavy metals, including Zn, Fe, Pb, Ni and Mn in the leaves of some plant species and leafy vegetables on the roadside in Karachi, Pakistan. These plant species (*Nerium oleander*, *F*. v*irens*, *Guaiacum officinale*, and *Ficus bengalensis)* accumulated the largest concentration of metals from roadside automobile pollution. Therefore, these plants can be used as a bio indicator in the future for roadside pollution [81]. Pirzada et al. [82] reported that the highest concentration of heavy metals was observed in *C*. *sativa* and *D*. *sissoo*. Thus, these species can be helpful for bioremediation of metals. Celik et al. [83] has observed a significant quantity of Zn, Mn, Fe, Ni, and Pb in leaves of *Robinia pseudo-acacia* L. and soil samples in Turkey. Tiwari et al. [84] noted that some plants were growing along roadsides can be used for phytoremediation of Fe and Mn. Heavy metals such as Pb, Mn, Zn and Ni in the roadside plants such as grasses and *Caesalpinia* species are accumulated in India [85–87]. These species could be used for bioindicators of heavy metals pollution on the roadside.

Ogbonna et al. [88] suggested that plants are related to some factors that can introduce some variation in the leaves for Pb and Ni. *Anarcadium occidentale* accumulated the high concentration of Pb and *Psidium guajava* absorbed the increased amount of Ni, which was the best indicator for urban air pollution [89]. In the current study, *A*. *nilotica* and *Z*. *mauritiana* were good bio-monitoring for Pb and Ni, respectively.

Jung et al. [90] conducted a study on heavy metals’ pollution and showed the highest concentration of Fe (8.73 ug/m^3^) near to subway station. The increased concentration of Fe occurred due to friction between the brake abrasion and wheel [91]. A similar study reported the heavy metal accumulation in wild plant species along the road [92]. The highest concentration of Zn was found in the *C*. *camphora*, and the leaves of *Populus euramevicana* [93]. In the present study, *A*. *nilotica*, *Z*. *mauritiana* and *C*. *procera* absorbed a higher amount of Zn, and *A*. *nilotica* accumulated a high amount of Fe. It is suggested that Fe plays a significant role in photosynthetic activity since it is accumulated in the chloroplast [94, 95].

The urban wild plants play a vital role in the environment like reducing the heat effect on the island and sink air pollutants [96]. Therefore vegetation and trees could be contributing to the control of air pollution and mitigate global warming [97].

Uka et al. [98] reported that the carotenoid content was lower for the leaf samples of four tree species, which were collected from the arterial road sites, and those species significantly differed at the control site except *Polyalthia longifolia* (p < 0.05). In the *Terminalia catappa* 0.11 mg/g of carotenoid content was noted at the Arterial road III. Additionally, *Polyalthia longifolia* has accumulated 0.17 mg/g of carotenoids at Arterial road I.

Many researchers estimated the reduced carotenoid content under roadside pollution [99, 100]. The reduction of carotenoid content at the New Lahore site, Nawababad site, and Fatehabad site induced the vehicular emission to reduce the pigments in the leaf samples [101]. The air emissions were transferred in the tissues through the stomata of leaves, which could be decreased the pigments in the leaf cells by the result of chloroplast denaturation [102]. Similarly, in other studies, reduced content of chlorophyll was observed [13, 103].

## Conclusion

The results showed that heavy metal pollution alters chemical composition of wild plants. *Z*. *mauritiana* is favorable for higher accumulation of Ni. Likewise, *R*. *communis* and *A*. *nilotica* accumulated higher amounts of Mn. For the control of Pb pollution, *Z*. *mauritiana* and *A*. *nilotica* proved suitable. Additionally, *R*. *communis* and *A*. *nilotica* are promising indicators for Zn and Fe. Overall, tested plant species reduced roadside pollution and can be used to control the heavy metal pollution from the roadside.
